The article "Modified Look-Locker Inverse-Recovery (MOLLI) Sequence of Quantitative Imaging in Dirty Magnetic Resonance Longitudinal Relaxation Time Diagnostic Value of GE Combined with Longitudinal Relaxation Time Quantitative Imaging for Myocardial Amyloidosis" was retracted in 2023. Reasons: signs of a paper mill; suspected computer-generated content; unreliable results or conclusions; lack of ethics approval or compliance.

# Modified Look-Locker Inverse-Recovery (MOLLI) Sequence of Quantitative Imaging in Dirty Magnetic Resonance Longitudinal Relaxation Time Diagnostic Value of GE Combined with Longitudinal Relaxation Time Quantitative Imaging for Myocardial Amyloidosis

**DOI:** 10.1155/2021/2800891

**Published:** 2021-10-19

**Authors:** Qun Lao, Wenping Xia, Jing Jin, Yuzhu Jia, Jianju Feng

**Affiliations:** ^1^Department of Radiology, Hangzhou Children's Hospital, Hangzhou, Zhejiang 310014, China; ^2^Department of Radiology, Yin Zhou Second Hospital, Ningbo, Zhejiang 315040, China; ^3^Department of Radiology, Tongde Hospital of Zhejiang Province, Hangzhou, Zhejiang 310012, China; ^4^Departments of Radiology, Zhuji Affiliated Hospital of Shaoxing University, Zhuji People's Hospital, Zhuji, Zhejiang 311800, China

## Abstract

The pathological changes of myocarditis include degeneration and necrosis of myocardial cells and infiltration of inflammatory cells in the myocardial interstitium, accompanied by obvious myocardial fibrosis. Myocardial fibrosis is a determinant of ventricular remodeling and an important indicator of the classification of clinical risk factors and has an important value in evaluating the prognosis of heart disease. Cardiac magnetic resonance (CMR) is the “gold standard” for evaluating the shape and function of the heart, and it can show the characteristic pathological changes of myocardial tissue. The traditional gadolinium imaging agent delays the enhanced sequence images to visually show the extent of the affected myocardial fibrosis, but it cannot effectively identify small focal fibrosis or widespread diffuse fibrosis. The CMR longitudinal relaxation time quantitative technique can directly measure the relaxation time (T1) determined by the myocardial tissue and does not depend on the signal strength of the reference tissue and can quantitatively analyze the affected myocardium. In this study, the initial and enhanced quantitative imaging techniques of CMR were used to measure the magnetic value of the myocardium in patients with myocarditis, to explore the diagnostic value of myocardial fibrosis, and to analyze the correlation between cardiac fibrosis and cardiac function.

## 1. Introduction

Myocardial fibrosis is a determinant of cardiac pathological remodeling caused by various cardiovascular diseases [1], is the pathological basis of abnormal cardiac mechanical function and electrical activity [2], and eventually leads to heart failure and increases patient mortality [3]. A large number of clinical studies have shown that [4, 5] the abnormal expansion of myocardial extracellular matrix (ECM) is reversible, and the therapeutic targets of some new research drugs are mainly for fibrosis or myocardial extracellular matrix expansion. Therefore, it is important to detect myocardial fibrosis and evaluate its extent or the degree of extracellular matrix expansion.

The article "Modified Look-Locker Inverse-Recovery (MOLLI) Sequence of Quantitative Imaging in Dirty Magnetic Resonance Longitudinal Relaxation Time Diagnostic Value of GE Combined with Longitudinal Relaxation Time Quantitative Imaging for Myocardial Amyloidosis" was retracted in 2023. Reasons: signs of a paper mill; suspected computer-generated content; unreliable results or conclusions; lack of ethics approval or compliance.

At present, clinical imaging tests commonly used in the clinic include echocardiography, cardiac CT, cardiac magnetic resonance (CMR), cardiovascular angiography, and myocardial radionuclide examination. What are the different examination methods? They have their advantages and values in the morphology, function, diagnosis, and differential diagnosis of myocardial lesions but they also have certain limitations. In recent years, CMR imaging technology has developed more and more rapidly, and clinical applications have become more and more widely used. It has become a routine examination method in cardiovascular centers and large hospitals. CMR has a good temporal and spatial resolution, arbitrary plane imaging, good repeatability, and other advantages. It can play cardiac morphology, function, myocardial tissue characteristics, and myocardial activity in heart disease. The “one-stop” inspection function has a unique value in the cause diagnosis, risk stratification, and prognosis judgment of cardiomyopathy, and it has become the most ideal noninvasive examination method for cardiomyopathy [6]. From a histological point of view, myocardial tissue includes intracellular components, intravascular components, and interstitial spaces. The extracellular matrix space of myocardium is surrounded by cardiomyocytes, capillaries, and nerves, and the gap is filled with the extracellular matrix. After activation of myofibroblasts, a series of processes lead to the deposition. According to the distribution, myocardial fibrosis can be divided into localized fibrosis and diffuse fibrosis. Localized fibrosis is more common in myocardial infarction. Diffuse fibrosis includes reactive fibrosis and interstitial fibrosis, and diffuse interstitial fibrosis is more seen in cardiomyopathy. CMR has unique advantages in the evaluation of myocardial histological features. In recent years, magnetic mapping technology has been gradually applied in clinical practice. In 2013, the Cardiac Magnetic Resonance Association and the European Radiological Society's Cardiac Magnetic Resonance Working Group issued an expert consensus to define magnetic mapping as a CMR method to directly measure the magnetic value of myocardial tissue before or after injection of the contrast agent. The signal strength of each pixel is encoded by the size of the pixel, and the parameter schematic diagram is drawn through computer postprocessing. According to previous reports, the gas magnetic mapping technology is divided into the initial magnetic (noncontrast agent or magnetic before injection of contrast agent) and the enhanced magnetic. Native magnetic value can noninvasively find the pathological changes of the heart such as changes in iron content because it does not require the injection of contrast agents and can be used in patients with severely impaired renal function. The magnetic value is obtained from a fitting curve of at least 6–10 time points, and the magnetic time needs to be measured in multiple cardiac cycles. At present, different manufacturers and equipment have different magnetic mapping sequences. Magnetic mapping can be implemented using inversion recovery (IR) or saturation recovery (SR) pulse sequences. The clinically used reversed recovery pulse sequence in the modified magnetic mapping technique is the MOLLI sequence. Under gating, a specific cardiac cycle (often at the end of diastole) is selected for data collection. An image is obtained every cardiac cycle, and a set of images can be obtained by continuously increasing the IR sequence of magnetics. MOLLI used preparation sequences to reconstruct images with different inversion times in one breath-hold in 17 cardiac cycles. The readout sequence adopts steady-state free precession (steady-state prediction, SSP), which can reduce the loss of the magnetization vector in the reverse recovery. The acquisition time is less than 200 ms, and there are few motion artifacts. It has high accuracy, repeatability, and spatial resolution [7–9]. It is currently the most commonly used in magnetic mapping technology, as shown in Figure 1. However, the MOLLI breath-holding time is longer, with heart rate dependence, and there are T2 dependence and other factors. The result of SSP reading is the recovery time magnetic, which is lower than the true value of myocardium. The magnetic value needs to be corrected.

The article "Modified Look-Locker Inverse-Recovery (MOLLI) Sequence of Quantitative Imaging in Dirty Magnetic Resonance Longitudinal Relaxation Time Diagnostic Value of GE Combined with Longitudinal Relaxation Time Quantitative Imaging for Myocardial Amyloidosis" was retracted in 2023. Reasons: signs of a paper mill; suspected computer-generated content; unreliable results or conclusions; lack of ethics approval or compliance.

In this study, segments accounted for 5.9%, mostly located in the inferior sidewalls. Previous work summarized the results of the multicenter study and speculated that the myocardial segmental magnetic value difference was not caused by different myocardial composition. The main reason why the MOLLI sequence affects the image quality classification is magnetically sensitive artifacts and respiratory and motion artifacts. The reading of MOLLI adopts an SSP sequence, which can produce magnetic sensitive artifacts similar to the movie sequence. 3.0 T magnetic resonance has higher signal-to-noise ratio and contrast-to-noise ratio, which can provide higher temporal and spatial resolution and shorten the scanning time. However, it is easy to produce a series of problems related to the unevenness of the main magnetic field and the RF field, such as the detuned resonance artifacts of the SSP sequence. But this does not fully reflect the extent of myocardial disease involvement. In this study, there was no statistically significant difference in apical image quality compared with the central and basal parts; and it is indicated that magnetic value can be measured and different sections of left ventricular myocardium can be obtained if the thickness of the apical myocardium is allowed. The magnetic value of the segment completely evaluates the fibrosis of all myocardium.

## 2. Research Methods and Objects

### 2.1. Materials and Methods

We collected 12 healthy volunteers who underwent CMR magnetic mapping technique scans between January 2015 and December 2016. The scanning sequence includes movie sequence and gadolinium contrast agent delayed enhancement; and magnetic mapping scanning includes more patients (before and after injection contrast agent scanning). The scan adopts the MOLLI sequence. After the scanning is completed, the time is automatically generated. The mentioned method was used to analyze the tapping parameters of the left ventricular myocardium. The mentioned portrayal and measurement are all done by Spin Lite software. Here, we use the Pearson correlation analysis to explore the correlation between each parameter and age. Finally, according to the coronary artery blood supply area, electrical currents were divided into three groups for comparison.

### 2.2. Health Conditions

According to the position statement of the European Society of Cardiology in 2015 [10], direct clinic mention (DCM) is defined as left ventricular (LV) or biventricular dilatation or systolic insufficiency and excludes abnormalities such as hypertension and valvular disease and causes large-scale contractile dysfunction coronary artery disease. Causes include genetic or nongenetic factors. The clinical manifestations are left ventricular or bilateral ventricular enlargement and reduced ventricular systolic function, with or without congestive heart failure and arrhythmia, and complications such as embolism and sudden death can occur, as shown in Figure 2. The condition is progressively worse, the prognosis is very poor, and death can occur at any stage of the disease. The 5-year mortality rate reported abroad is 50%, and the domestic epidemiological survey found that the 5-year mortality rate is 80%. DCM ranks third among common causes of heart failure and ranks first among heart transplants [11]. According to Laplace's law, increased intraventricular wall tension leads to increased oxygen consumption and decreased myocardial contractile function. Decreased cardiac function forms a vicious cycle, progressive ventricular dilation, and relative thinning of the wall, and enlargement of the ventricular sphere eventually leads to ventricular remodeling, as well as microvascular damage, abnormal myocardial blood flow, and left ventricular block; and abnormal right ventricular pacing is also exacerbated. CMR imaging technology has developed more and more rapidly, and clinical applications have become more and more widely used. It has become a routine examination method in cardiovascular centers and large hospitals. CMR has a good temporal and spatial resolution, arbitrary plane imaging, good repeatability, and other advantages. It can play cardiac morphology, function, myocardial tissue characteristics, and myocardial activity in heart disease.

The article "Modified Look-Locker Inverse-Recovery (MOLLI) Sequence of Quantitative Imaging in Dirty Magnetic Resonance Longitudinal Relaxation Time Diagnostic Value of GE Combined with Longitudinal Relaxation Time Quantitative Imaging for Myocardial Amyloidosis" was retracted in 2023. Reasons: signs of a paper mill; suspected computer-generated content; unreliable results or conclusions; lack of ethics approval or compliance.

The process of ventricular remodeling eventually leads to direct clinical mention (DCM). The magnetic mapping technique can improve the sensitivity of CMR diagnosis of myocarditis and can be used as an effective means for the assessment of myocarditis condition and efficacy. The fibers of DCM are tandem hyperplasia and eccentric hypertrophy of the heart, the heart is significantly enlarged, the wall thickness is normal or slightly thickened, and the ventricles on both sides are excessively trabeculated. The left ventricular myocardial thickness is increased or thinned due to the enlargement of the heart cavity. Occasionally a subendocardial thrombus can be seen in the heart cavity. DCM has no specific histological manifestations and cardiomyocytes vary in size, cytoplasmic vacuolation, abnormal nuclei, and abnormal chromatin arrangement [12]. Alternative fibrosis in the middle layer can extend from the interventricular septum to the free wall or diffuse fibrosis. Some inflammatory DCM may have focal lymphocyte infiltration [13]. There are often thickened fibers under the endocardium. The cause of fibrosis in the interventricular septal muscle is unknown. Myocardial fibrosis leads to increased wall rigidity, reduced ventricular contraction, and diastolic function, leading to hemodynamic changes. Myocardial fibrosis can also cause fatal arrhythmias, leading to serious complications. The myocardial interstitial fibrosis in DCM patients is extensive, and the extracellular matrix is enlarged. The gadolinium contrast agent is concentrated outside the cell, showing delayed enhancement. CMR's problem has certain advantages for the detection of early moderate myocardial fibrosis. The problem may be a potential tool for predicting the risk stratification of DCM cardiac risk events.

The degree of myocardial diffuse fibrosis in patients with hypertensive heart disease and left ventricular hypertrophy is higher than that in simple hypertensive heart disease group and normal control group, and an electrical current is positively correlated with left ventricular myocardial mass index. It has a significant correlation with cardiovascular mortality, sudden cardiac death, and heart failure hospitalization rates. It is an independent predictor of cardiovascular death and heart transplant events. But myocardial diffuse fibrosis, lack of fibrosis, and normal myocardium, leading to mild fibrosis lesions, cannot show these problems [13]. Studies have confirmed [14] that the distribution of fibrotic tissue in DCM patients has a high degree of consistency with delayed enhancement sites, mainly manifested as intermuscular wall enhancement, which is related to poor prognosis, as shown in Figure 3. Fifty percent of patients present with negative performance. Coronary artery-negative myocardium [15] is likely to have undergone diffuse fibrosis in pathology. The negative coronary artery does not rule out myocardial disease. Previous studies [16] have shown that coronary artery can be associated with adverse cardiac events or arrhythmias but not with cardiac function. A study by Reiter et al. [17] has shown that, in patients with dilated cardiomyopathy, the value of Natal is related to left ventricular remodeling and myocardial contractile function. Stromp et al. [18] performed CMR examination and endocardial biopsy on 47 patients with cardiomyopathy, and 13 normal controls were used as the control group. The results showed that the magnetic values of the control group were greater than those with a negative coronary artery or accompanied by the obvious coronary artery.

The article "Modified Look-Locker Inverse-Recovery (MOLLI) Sequence of Quantitative Imaging in Dirty Magnetic Resonance Longitudinal Relaxation Time Diagnostic Value of GE Combined with Longitudinal Relaxation Time Quantitative Imaging for Myocardial Amyloidosis" was retracted in 2023. Reasons: signs of a paper mill; suspected computer-generated content; unreliable results or conclusions; lack of ethics approval or compliance.

Magnetic value is negatively correlated with histological fibrosis, similar to the above study results; and magnetic value can be used to noninvasively assess diffuse endocardial fibrosis in patients with cardiomyopathy. Schaefer et al.'s [19] study shows that the electrical current of DCM patients is higher than that of normal people, and it is related to cardiac function [20]. 45 cases of early DCM (mild cardiac function impairment and enlarged heart cavity, between 45% and 55%), 29 cases of DCM (impaired cardiac function, EF < 45% and enlarged heart chambers), and 56 healthy controls underwent CMR examination, showing that early DCM electrical current (25% ± 4%) and DCM electrical current (27% ± 3%) increased, higher than the healthy control (23% ± 3%), and there was a statistical difference (>0.05). Four patients with DCM underwent endocardial biopsy, and there was a significant correlation between CVF and electrical current (*r* = 0.85, *p*=0.01), indicating that the early DCM electrical current can be increased, and the electrical current value can be reflected myocardial collagen deposition. Electrical current can be used as a noninvasive method and quantitative tool for the detection of myocardial fibrosis and can be used to monitor the response and risk stratification of DCM treatment.

The article "Modified Look-Locker Inverse-Recovery (MOLLI) Sequence of Quantitative Imaging in Dirty Magnetic Resonance Longitudinal Relaxation Time Diagnostic Value of GE Combined with Longitudinal Relaxation Time Quantitative Imaging for Myocardial Amyloidosis" was retracted in 2023. Reasons: signs of a paper mill; suspected computer-generated content; unreliable results or conclusions; lack of ethics approval or compliance.

### 2.3. Complications

The tissue characteristics of myocarditis include myocardial edema, hyperemia, and necrosis or fibrosis. The subendocardial biopsy is an important method to diagnose myocarditis, but it may cause complications or adverse consequences, and the tissue intensity can be summarized as in Figure 4. Patients with acute myocarditis have increased water content of myocardial cells due to inflammation. Myocardial ischemia leads to changes in the distribution of sodium and potassium inside and outside the cell, affecting free proton movement, resulting in a significant increase in magnetic relaxation time compared with normal people. Studies have shown that the accuracy of the magnetic mapping technique in the diagnosis of myocarditis is significantly higher than the “Lake” diagnostic criteria. Other studies have shown that the Postel value and electrical current value can identify the potential myocardial damage in the “normal” myocardium of children with myocarditis. The other 25 patients with acute myocarditis and normal controls underwent black blood mapping and coronary artery scans, respectively, and it was found that the magnetic value of patients with acute myocarditis was significantly higher than that of the control group, and there was a statistical difference. Myocarditis sensitivity (91.5%) and accuracy (90.4%) were significantly higher than black blood T2 sequence (50.3% and 64.2%) and coronary artery sequence (73.1% and 83.0%). The specificity (89.2%) is lower than acute myocarditis (96.3%) and higher than the black blood sequence (88.5%) and has a good diagnostic value for acute myocarditis, especially. It is a diffuse lesion and a small focal lesion, which is similar to the results of Ferreira and other studies, and the quantitative advantage is more significant.

Tapping can be used to quantitatively evaluate the degree of myocardial diffuse fibrosis in patients with hypertension and heart disease, especially the magnetic value and electrical current value. The degree of myocardial diffuse fibrosis in patients with hypertensive heart disease and left ventricular hypertrophy is higher than that in simple hypertensive heart disease group and normal control group, and an electrical current is positively correlated with left ventricular myocardial mass index. Patients with hypertensive heart disease and left ventricular hypertrophy with diastolic dysfunction have higher magnetic and electrical current values than patients with hypertensive heart disease and hypertensive heart disease and left ventricular hypertrophy without cardiac dysfunction, suggesting that the myocardial diffuse interstitial fibers as shown in Figure 5 are more serious. Electrical current can also identify myocardial fibrosis in patients with hypertension and heart disease at an early stage and is an independent predictor of arrhythmia (atrial fibrillation), diastolic heart failure, and death in patients with hypertension and heart disease. The pathological change is the deposition of amyloid in the extracellular space, which leads to an increase in the volume of the extracellular space. After enhanced scanning, gadolinium is deposited in the enlarged extracellular space, and delayed enhancement may occur. The typical acute myocarditis manifestations are as follows: (1) acute myocarditis diffuse full-thickness subendocardial or transmural enhancement; (2) contrast medium being cleared quickly from the blood pool, and the heart cavity having dark blood pool performance; and (3) magnetic medium scan.

The article "Modified Look-Locker Inverse-Recovery (MOLLI) Sequence of Quantitative Imaging in Dirty Magnetic Resonance Longitudinal Relaxation Time Diagnostic Value of GE Combined with Longitudinal Relaxation Time Quantitative Imaging for Myocardial Amyloidosis" was retracted in 2023. Reasons: signs of a paper mill; suspected computer-generated content; unreliable results or conclusions; lack of ethics approval or compliance.

The myocardium is inhibited earlier than the heart cavity. Not only can acute myocarditis be used for diagnosis but also it reflects the distribution of amyloid, suggesting that the myocardial load of amyloid is an independent prognostic factor. The characteristic enhancement pattern of acute myocarditis can also be distinguished from scars of ischemic cardiomyopathy and myocardial fibrosis of nonischemic cardiomyopathy. The coronary artery's acute myocarditis also tends to develop from normal no enhancement to subendocardial enhancement to transmural enhancement. Therefore, the enhancement pattern changes greatly, and the typical performance occurs in the late stage of the disease, and early lesions can be without acute myocarditis. Many patients with immune light chain amyloidosis (ALCH) have kidney involvement at the same time and cannot perform enhanced scans. The initial magnetic mapping technique does not require contrast agents and can be used for the detection of amyloidosis infiltration degree and efficacy. The electrical current value is significantly higher than that of cardiomyopathy patients and normal control groups, and the distribution of electrical current and acute myocarditis segments is consistent. The value of Natl can diagnose coronary artery. Here we found that the threshold value of AL type is 1020 ms and the diagnostic accuracy is 92%, which has a significant correlation with systolic and diastolic dysfunction. The magnetic value with significantly improved accuracy can reflect the cardiac amyloid load. In the study, the coronary artery's national magnetic value is higher than that of normal volunteers. Our research shows that the magnetic value is about 16% higher than normal and is related to cardiac systolic and diastolic function. Native value is more sensitive to early changes of the disease and prolonged magnetic value, and increased electrical current precedes changes in cardiac hypertrophy. The increase of magnetic value can reflect the severity of the disease and myocardial load. The magnetic value can also be used for treatment monitoring. Studies such as paintings have found that the left ventricular myocardial mass (LVM) of 7 patients who took green tea extract for 12 months decreased, accompanied by a decrease in magnetic value and electrical current, suggesting a decrease in myocardial load of amyloid. Studies have shown that electrical current >0.45 has a significant correlation with mortality (>4.41). Electrical current can be used as a biological indicator for predicting the prognosis of AL.

The article "Modified Look-Locker Inverse-Recovery (MOLLI) Sequence of Quantitative Imaging in Dirty Magnetic Resonance Longitudinal Relaxation Time Diagnostic Value of GE Combined with Longitudinal Relaxation Time Quantitative Imaging for Myocardial Amyloidosis" was retracted in 2023. Reasons: signs of a paper mill; suspected computer-generated content; unreliable results or conclusions; lack of ethics approval or compliance.

## 3. Clinical Manifestations

### 3.1. Extracellular Matrix and Myocardial Fibrosis

Myocardial fibrosis is a determinant of cardiac pathological remodeling caused by various cardiovascular diseases, is the pathological basis of abnormal cardiac mechanical function and electrical activity, and eventually leads to heart failure and increases patient mortality. A large number of clinical studies have shown that the abnormal expansion of the myocardial extracellular matrix is reversible, so the therapeutic targets of some new research drugs are mainly aimed at fibrosis or myocardial extracellular matrix expansion. Therefore, it is important to detect fibrosis and evaluate the extent of myocardial fibrosis or the degree of expansion of the extracellular matrix. Myocardial tissue includes three components: (1) cellular components, including cardiomyocytes, fibroblasts, epithelial cells, smooth muscle cells; (2) intravascular components, namely, blood; and (3) interstitial space, except for cells and vascular cells. The outer matrix is partially filled. In normal myocardial tissue, myocardial cells are closely packed, and there is little extracellular matrix. The extracellular interstitial space is a complex, mesh-like three-dimensional space surrounded by cardiomyocytes, capillaries, and nerves; it is mainly composed of collagen scaffolds, of which the first situation is 85% and the second is 11%, as shown in Figure 6. It is clinically suspected that the increase of electrical current during the coronary artery is early. Period involvement is more sensitive than acute myocarditis, and the change in electrical current is more obvious than magnetic value, which can be used as a new indicator to assess the severity of the coronary artery. Besides, it surrounds cardiomyocytes and the coronary artery between muscles maintains the dynamic balance, support, and integrity of the myocardial structure and has the function of preventing the myocardial fibers from slipping and supporting the mechanical function of the myocardial tissue; there are various proteins and information molecules (signaling molecules) in the interstitial space. The intracellular scaffold proteins and intercellular proteins establish links and transmit biochemical signals. Extracellular matrix affects myocardial fibrosis and secondary cardiac tissue structure and cardiac function changes. After activation of myofibroblasts, a series of processes lead to the deposition, mainly the formation of thick and ductile collagen, which forms various forms of fibrosis visible to the naked eye, resulting in abnormal heart function or conduction.

The article "Modified Look-Locker Inverse-Recovery (MOLLI) Sequence of Quantitative Imaging in Dirty Magnetic Resonance Longitudinal Relaxation Time Diagnostic Value of GE Combined with Longitudinal Relaxation Time Quantitative Imaging for Myocardial Amyloidosis" was retracted in 2023. Reasons: signs of a paper mill; suspected computer-generated content; unreliable results or conclusions; lack of ethics approval or compliance.

The extracellular matrix is damaged under the action of matrix magnetic metalloproteinases (MMPs). The relative levels of tissue inhibitors of metalloproteinases determine the rate of damage. Inflammatory cells and other cytokines also affect the process of myocardial fibrosis. Myocardial fibrosis includes alternative fibrosis and interstitial fibrosis, and the former can be seen in patients with myocardial cell necrosis or myocardial infarction; and the latter can be seen in nonischemic cardiomyopathies, such as sarcoidosis, myocarditis, and chronic renal insufficiency. Interstitial fibrosis can be diffuse, including reactive fibrosis and infiltrating interstitial fibrosis. Reactive fibrosis is seen in aging, high blood pressure, and diabetes. Myocardial fibrosis is a complex process that leads to aggregation/expansion of extracellular matrix and stiff ventricular wall, affects diastolic function, and ultimately damages cardiac contractile function and also affects normal cell activities such as myocardial electrophysiology.

### 3.2. Myocardial Fibrosis Evaluation Tool

#### 3.2.1. Contrast Agent-Delayed Strengthening

An endocardial biopsy is the “gold standard” for diagnosing myocardial fibrosis, but it is an invasive test and may have sampling errors, which limits clinical application. Acute myocarditis is considered to be the “gold standard” for noninvasive detection of myocardial focal fibrosis. The gadolinium contrast agent is an extracellular space contrast agent, which cannot enter the cell through the intact cell membrane. Its function is to shorten the magnetic relaxation time of the tissue. Myocardial fibrosis deposits in extracellular interstitial collagen, causing the body to expand. A gadolinium contrast agent is deposited and concentrated in the extracellular matrix, and the capillary density in the affected area is reduced, and the outflow rate is slowed which shortens the relaxation time of myocardial fibrosis magnetic and is more obvious than the normal myocardial shortening. Delayed scanning adopts magnetic-weighted inversion recovery sequence imaging. The inversion time is artificially set so that the normal myocardial signal is 0 (black), and the fibrotic tissue is a local high signal (showing white), which is in obvious contrast with the surrounding normal tissue. Acute myocarditis is the “gold standard” for imaging scars and fibrosis, especially for focal fibrosis, which has good repeatability. Acute myocarditis of different diseases has different manifestations of myocardial fibrosis, so it can be prompted and identified. However, acute myocarditis also has corresponding problems; and the coincidence rate can be realized into continuous growth, as shown in Figure 7. The pathogenesis of DCM is caused by stress load, volume load, and neurohormonal hyperresponsiveness, leading to apoptosis, death, and fibrosis of myocardial cells, and myocardial cells are rarely regenerated and renewed. The myocardium is damaged and the cytoskeleton is dissolved, and the ventricular cavity is enlarged. In the early stage of the disease, acute myocarditis's performance characteristics can indicate the faults, but, in the late stage of the disease, acute myocarditis is diffusely distributed and the performance is not specific. It is difficult to identify the cause. Currently, acute myocarditis is mainly judged visually, and there is no unified threshold; and it depends on fibrosis and surrounding normal tissues. Compared with the signal, the boundary of the lesion area is generally not clear enough. There is no objective standard when judging the edge of acute myocarditis and measuring the range of acute myocarditis. When the window width and window position are changed, the range also changes, especially in ischemic cardiomyopathy. Before the acute myocarditis scan, you must first perform a sequence scan to find the appropriate magnetic time for normal myocardial tissue suppression.

The article "Modified Look-Locker Inverse-Recovery (MOLLI) Sequence of Quantitative Imaging in Dirty Magnetic Resonance Longitudinal Relaxation Time Diagnostic Value of GE Combined with Longitudinal Relaxation Time Quantitative Imaging for Myocardial Amyloidosis" was retracted in 2023. Reasons: signs of a paper mill; suspected computer-generated content; unreliable results or conclusions; lack of ethics approval or compliance.

If the myocardium is diffusely fibrotic, the scanner will mistakenly think that the fibrotic myocardium is normal and incorrectly set the reverse. At the time of transfer, acute myocarditis will display diffuse fibrosis lesions as black, causing its false normalization. However, it will not display diffuse fibrosis, resulting in missed diagnosis, such as diseases with volume load or pressure load overload. There is no abnormal signal delayed enhancement, abnormal heart changes cannot be ruled out. It can be seen that there is no optimal threshold for acute myocarditis on CMR which can well reflect myocardial fibrosis. The signal strength of acute myocarditis cannot accurately identify the type of fibrosis. In patients with renal dysfunction, the gadolinium contrast agent will aggravate the change of renal fibrosis and increase the occurrence of contrast agent nephropathy and cannot be enhanced. Therefore, the quantitative technique based on the inherent properties of the tissue and the direct measurement of the magnetic value and the electrical current technique of extracellular interstitial volume fraction have become research hotspots in recent years. Such techniques can more sensitively detect early and diffuse myocardial fibrosis and improve the diagnostic efficacy of CMR. In October, our working group put forward the consensus of quantitative evaluation of magnetic mapping and extracellular mesenchymal volume fraction (extracellular, fractional, electrical current).

#### 3.2.2. Magnetic Mapping Sequence

After using inversion recovery (IR) or saturation recovery (SR) pulse sequence scanning, the magnetic mapping parameter map of the heart is generated by each pixel in the magnetic value coding map. In the reverse recovery sequence, the magnetic mapping technology and the improved Look-Locker magnetic mapping technology are commonly used. The Loop-Locker magnetic mapping technology periodically applies a series of low flip angle (<35°) RF pulses to generate gradient echoes. After the magnetization vector is reversed, it uses gradient echoes to read out after each RF pulse. The MR signal quantifies the magnetic value according to the rate of change of the signal amplitude. This sequence can be acquired multiple times under multiple magnetic values, and the imaging speed is fast. The disadvantage is that the gradient echo readout signal causes the inversion recovery curve to change which may lead to inaccurate magnetic measurement and is not suitable for a beating heart. MOLLI technology utilizes balanced steady-state precession (SSP) sequence to read out the signal which can reduce the loss of magnetization vector during reverse recovery and has a smaller impact on the longitudinal magnetization vector recovery curve and can obtain a higher signal-to-noise ratio. From this result, we can use mapping-gating to perform selective image acquisition at the end of diastole, effectively reducing the impact of a heartbeat on image acquisition. The sequence generates a data set that increases the number of samples in the relaxation curve, thereby making the measurement accuracy of magnetic higher in 3.0 T MRI compared to the CT and 1.5 T MRI mappings as shown in Figure 8. The scan was completed within 17 cardiac cycles, and 5 single acquisitions were performed with 3 cardiac cycles without data acquisition between each acquisition. The initial magnetic time is the time from the application of the inversion pulse to the acquisition of the first image in k-space. The effective magnetic time is the length of the cardiac cycle from the beginning of the first image acquisition at the initial time.

The article "Modified Look-Locker Inverse-Recovery (MOLLI) Sequence of Quantitative Imaging in Dirty Magnetic Resonance Longitudinal Relaxation Time Diagnostic Value of GE Combined with Longitudinal Relaxation Time Quantitative Imaging for Myocardial Amyloidosis" was retracted in 2023. Reasons: signs of a paper mill; suspected computer-generated content; unreliable results or conclusions; lack of ethics approval or compliance.

MOLLI can collect all tapping data of a single layer of the heart in a breath-holding process. The collection time is less than 200 ms, and there are few motion artifacts. High accuracy, repeatability, and spatial resolution are currently the most commonly used technologies. However, breath-holding time is longer. With heart rate dependence, there are factors such as dependence, magnetization transfer, inversion efficiency, and loss of magnetization vector. The result of SSP reading is the recovery time magnetic, which is lower than the true value of myocardium. Therefore, magnetic mapping needs to be corrected. Common saturation recovery (SR) sequence acquisition method is saturation recovery single-shot acquisition, which is not subject to the measurement within 10 cycles of a heartbeat cycle, and the A-frame measurement is performed within 10 cycles. The SSP sequence read signal is not affected by the loss of the longitudinal magnetization vector and is also not affected by the absolute magnetic value, heart rate, and flip angle. It is more accurate than MOLLI, but the signal noise is lower and the artifacts are more than the latter. Therefore, by this method, the accuracy is reduced.

## 4. Simulation Experiment and Result Analysis

### 4.1. Longitudinal Relaxation Time

Magnetic mapping technology includes the initial (before enhancement) magnetic mapping and enhanced magnetic mapping. The initial magnetic mapping is to measure the magnetic value of the myocardium by scanning the noninjected contrast agent. This technique is highly repeatable and is not affected by contrast injection. It is suitable for patients with renal insufficiency or contrast allergy. After enhancement, time-mapping is usually injected with a contrast agent at a dose of 0.15–0.220 mm/kg. After 15–20 minutes of injection, an image is collected to measure the myocardial posttime value, but the posttime value is affected by a variety of factors, such as contrast agent dose, concentration, injection rate, and collection time after injection. The increase in the value could be found in the following factors: (1) cell necrosis caused by myocardial injury or myocardial inflammation and (2) myocardial amyloidosis or fibrosis (myocardial infarction scar, hypertrophic cardiomyopathy, dilated cardiomyopathy, etc.). The decrease in the value is seen in myocardial fat infiltration (such as Anderson-Fabry disease) and myocardial iron deposition disease. However, the magnetic value is dependent on heart rate. Due to the cardiac cycle, the magnetic value in diastole is slightly higher than that in systole, which may be due to the difference in myocardial blood volume between systole and diastole. The magnetic value is also affected by the myocardial segment. Here, we found that the apex is larger than the basal and central native measurements, which may be related to the thinner wall of the apex and the greater proportion of extracellular interstitial. Also, it may be related to the apical image being more susceptible to partial volume effect interference. Moreover, we summarized the results of the multicenter study and speculated that the difference in myocardial segmental magnetic value was not caused by different myocardial composition. But the magnetic field uniformity could be reached into the highest point in a certain time as shown in Figure 9. When there is a difference between the measurement segments, it is necessary to consider the existence of these objective factors, rather than direct judgment as myocardial injury. Gender and age are also physiological factors that affect the magnetic value, but the conclusion is not uniform.

The article "Modified Look-Locker Inverse-Recovery (MOLLI) Sequence of Quantitative Imaging in Dirty Magnetic Resonance Longitudinal Relaxation Time Diagnostic Value of GE Combined with Longitudinal Relaxation Time Quantitative Imaging for Myocardial Amyloidosis" was retracted in 2023. Reasons: signs of a paper mill; suspected computer-generated content; unreliable results or conclusions; lack of ethics approval or compliance.

### 4.2. Extracellular Matrix Volume Fraction

The magnetic value is affected by the strength of the magnetic field and the accuracy of the measurement method, and these effects may exceed the difference between the normal myocardium and diseased myocardium, making it difficult to directly compare the value under different conditions. Moreover, the magnetic value includes two parts: the interstitial part and cardiomyocytes part. The electrical current of the myocardium reflects the volume fraction of the myocardial tissue that is not occupied by the cells. The electrical current value can be calculated by adjusting the myocardial value and the magnetic value of the myocardium through the blood cell volume, and the electrical current map is generated accordingly. Electrical current measures the space occupied by extracellular interstitium and is correlated with the collagen volume fraction (collapse evolution, CVF).

The typical characteristics of acute myocarditis in HCM patients are patchy or large acute myocarditis between muscles, which are common in the anterior wall, the right ventricular insertion part of the base, the anterior septum, and the area of myocardial hypertrophy, and nonhypertrophic areas appear. In the case of noninvasive disease and edema, electrical current can be used as a biological marker of myocardial fibrosis. The electrical current value is less affected by changes in magnetic field strength. It is affected by the dose of contrast agent, delay time, glomerular filtration rate, hematocrit, and body fat content. Contrast agent injection methods include continuous intravenous infusion and a single bolus injection of contrast agent. From this, we can achieve a dynamic equilibrium state of distribution between plasma and interstitial. We compared two injection methods of normal volunteers, and the difference was not statistically significant. The accuracy of MRI in the first sample is higher than the second value and the third value as shown in Figure 10. But the individual varies greatly. Here we found that electrical current in females is higher than that in males. If itself is high, there are statistical differences, which may be inherent. Most of the current literature also supports this view. An electrical current map can intuitively provide the electrical current value of each pixel, which significantly shortens the measurement time compared to manual measurement, but it may affect the measurement due to poor registration and image correction.

The article "Modified Look-Locker Inverse-Recovery (MOLLI) Sequence of Quantitative Imaging in Dirty Magnetic Resonance Longitudinal Relaxation Time Diagnostic Value of GE Combined with Longitudinal Relaxation Time Quantitative Imaging for Myocardial Amyloidosis" was retracted in 2023. Reasons: signs of a paper mill; suspected computer-generated content; unreliable results or conclusions; lack of ethics approval or compliance.

### 4.3. Clinical Application

The study of the magnetic value before and after infarction found that the initial magnetic mapping can detect myocardial infarction; and the acute myocardial infarction native value (1197 ± 76 ms) is higher than the old myocardial infarction native value (1060 ± 61 ms). Magnetic mapping sensitivity and specificity for the diagnosis of acute myocardial infarction can reach 96% and 91%, which is more sensitive than second mapping. Compared with acute myocardial infarction, the abnormal area of the magnetic value of old myocardial infarction is closer to the range of acute myocarditis display infarction and has a good consistency. However, the abnormal area of magnetic value is larger than the range of acute myocarditis, suggesting that the mapping can be used. Screening for acute myocardial infarction is not suitable for assessing infarct size. Magnetic mapping can quantify the value of myocardial edema of acute myocardial infarction (AMI), reflecting the scope of edema. Magnetic mapping technique combined with acute myocarditis can accurately determine the inversion of myocardial infarction. The value of mapping can also identify the microvascular obstruction. The microvascular area is higher than the distal myocardium but lower than the infarcted myocardium. Magnetic mapping technology can evaluate the degree and severity of the myocardial injury. Here, by using acute myocarditis and mapping as a tool, it was found that native magnetic is significantly related to the severity of the myocardial injury, and magnetic value can predict the recovery of cardiac function. Calculating electrical currents can also accurately diagnose the range of myocardial infarction. The electrical current range of normal myocardium is 24%. In another part, the electrical current of patients with acute myocardial infarction at 1 week was 58.5% ± 7.6%. Our research shows that the electrical current of old myocardial infarction reached 68.5% ± 8.6%. After myocardial infarction, apoptosis is widespread in the infarct area and the noninfarct area. The myocardial cell apoptosis in the noninfarct area and the late ventricular remodeling are mutually causal, leading to the continuous deterioration of cardiac function.

The article "Modified Look-Locker Inverse-Recovery (MOLLI) Sequence of Quantitative Imaging in Dirty Magnetic Resonance Longitudinal Relaxation Time Diagnostic Value of GE Combined with Longitudinal Relaxation Time Quantitative Imaging for Myocardial Amyloidosis" was retracted in 2023. Reasons: signs of a paper mill; suspected computer-generated content; unreliable results or conclusions; lack of ethics approval or compliance.

The increase of electrical current indirectly suggests that the apoptosis and displacement of the noninfarct area may be related to the mechanism of myocardial remodeling in the noninfarct area. Studies also show that magnetic value in the noninfarct area is heart failure after myocardial infarction. Independent variables are related to cardiac adverse events and death. Although acute myocarditis is still the most important method for detecting acute and old myocardial infarction, magnetic mapping and electrical current can further quantitatively evaluate noninfarct myocardium and the area around the infarct from different angles, which can provide more pathophysiology for the diagnosis and treatment of myocardial infarction information. The new guideline of the European Society of Cardiology in 2014 expanded the definition of hypertrophic cardiomyopathy, which can be regarded as the newfound when the patient has left ventricular wall thickening and increased cardiac load as a nonindependent pathogenic factor. This definition includes not only cardiac muscle. Autosomal dominant genetic diseases caused by mutations in globulin genes also include metabolic and neuromuscular genetic diseases, chromosomal inheritance, and genetic syndromes, as well as aging and amyloidosis. Hypertrophic cardiomyopathy is characterized by ventricular wall hypertrophy, mainly involving the left ventricle. The incidence is about 1/500 and the case fatality rate is nearly 1/1000, which is one of the main causes of sudden death in young adults. Hypertrophic histological cardiomyopathy showed that myocardial cells were hypertrophic and the nuclei were abnormal under the microscope. They were arranged in an irregular, chaotic, herringbone pattern. In asymmetric ventricular septal hypertrophic cardiomyopathy, the increase in myocardial cells also exacerbates ventricular septal hypertrophy. The abnormalities of extracellular interstitial include interstitial fibrosis and alternative fibrosis; in particular, plexiform fibrosis can be seen in the chaotically arranged areas. Interstitial fibrosis can be seen around normal or abnormal cardiomyocytes; alternative fibrosis can extend to areas where cardiomyocytes are missing.

The article "Modified Look-Locker Inverse-Recovery (MOLLI) Sequence of Quantitative Imaging in Dirty Magnetic Resonance Longitudinal Relaxation Time Diagnostic Value of GE Combined with Longitudinal Relaxation Time Quantitative Imaging for Myocardial Amyloidosis" was retracted in 2023. Reasons: signs of a paper mill; suspected computer-generated content; unreliable results or conclusions; lack of ethics approval or compliance.

Occasionally, there are abnormalities in the intermural coronary arteries, the development of small intermural arteries, the thickening of the intima, and intima with a structural disorder of the intima. Hypertrophic cardiomyopathy fibrosis may be related to two reasons: (1) model caused by abnormal myocardial cells, as well as interstitial and plexiform fibrosis caused by histopathological reactions, and (2) narrowed coronary artery lumen stenosis caused by small abnormalities. Chronic infarction impairs hypertrophic myocardial perfusion and reduces coronary reserve capacity. Previous studies have shown that the interventricular septal area is more common to the intermural arterioles, and the areas with obvious fibrosis are more common than the areas with no or light fibrosis. This result indicates the stage of disease progression. End-stage acute myocarditis patients have a wider range than those who preserve cardiac function. Acute myocarditis is associated with the occurrence of ventricular arrhythmias. Extensive acute myocarditis is associated with an increased risk of sudden cardiac death (SCD) and decreased end-stage systolic function. Acute myocarditis is a risk factor for sudden cardiac death. Acute myocarditis is expected to provide a basis for the risk stratification of SCD and guide implantable cardioverter-defibrillator (ICD) implantation treatment. Histopathologically, the acute myocarditis region reflects alternative fibrosis and end-stage hypertrophic cardiomyopathy fibrosis. Acute myocarditis generally does not appear in the mild fibrosis zone, because the signal in the small fibrosis zone can be completely suppressed. Hypertrophic cardiomyopathy fibrosis is common and the degree of fibrosis of the affected myocardium is different through 48 hypertrophic cardiomyopathy patients and 18 normal controls. Magnetic mapping technique can be used to determine the severity of myocardial fibrosis in hypertrophic cardiomyopathy patients. The evaluation shows that there are different degrees of fibrosis in the surrounding area of acute myocarditis, suggesting that lesions in the early stage of fibrosis can be found. Native magnetic value is valuable for detecting this part of the anomaly without acute myocarditis, and the electrical current value is significantly higher than normal control. We analyzed the results of magnetic mapping's assessment of myocardial fibrosis with the results of high-throughput gene sequencing and endocardial biopsy and found that the mapping values of hypertrophic cardiomyopathy-related gene carriers were significantly shortened after a delay. The decrease of the value is significantly related to the patient's left ventricular diastolic dysfunction, suggesting that the diffuse fibrosis measured by mapping can be used as a powerful tool to link the phenotype and genotype of the patient.

The article "Modified Look-Locker Inverse-Recovery (MOLLI) Sequence of Quantitative Imaging in Dirty Magnetic Resonance Longitudinal Relaxation Time Diagnostic Value of GE Combined with Longitudinal Relaxation Time Quantitative Imaging for Myocardial Amyloidosis" was retracted in 2023. Reasons: signs of a paper mill; suspected computer-generated content; unreliable results or conclusions; lack of ethics approval or compliance.

## 5. Conclusion

This shows that the application of magnetic mapping and electrical current techniques in CMR examination can improve the accuracy of coronary artery diagnosis, quantify amyloid load, distinguish coronary artery types, and predict prognosis. In summary, magnetic mapping technology and electrical current technology can detect early and can quantitatively evaluate the lesions. It has good application prospects in the diagnosis, risk assessment, efficacy, and prognosis evaluation of various myocardial diseases. However, magnetic mapping technology and electrical current technology are affected by many factors. At present, there is a lack of a unified normal reference value. Moreover, large-scale and multicenter research is still required.

In the future, electrical current can be used as a biological marker of myocardial fibrosis. The electrical current value is less affected by changes in magnetic field strength. It is affected by the dose of contrast agent, delay time, glomerular filtration rate, hematocrit, and body fat content.

## Figures and Tables

**Figure 1:** Magnetic mapping technology for the modular mapping.

**Figure 2:** Health conditions measured by a series of imaging processes.

**Figure 3:** Distribution of the fibrotic tissue in DCM patients.

**Figure 4:** Tissue characteristics of myocarditis based on the MRI energy.

**Figure 5:** Hypertensive heart disease and left ventricular hypertrophy with diastolic dysfunction.

**Figure 6:** Collagen scaffolds in the mesh-like three-dimensional space.

**Figure 7:** Coincidence rate under a continuous observation time.

**Figure 8:** Compatibility of magnetic measurement in the MRI and CT mappings.

**Figure 9:** Magnetic value-respective hip angle changes with time.

**Figure 10:** Accuracy of MRI value in the different samples.

## Data Availability

The data used to support the findings of this study are available from the corresponding author upon request.
